RETRACTED

# CAMPO Precision128 Max ENERGY Spectrum CT Combined with Multiple Parameters to Evaluate the Benign and Malignant Pleural Effusion

**DOI:** 10.1155/2021/5526977

**Published:** 2021-02-26

**Authors:** Tianyu Zhang, Cuicui Wu, Zhongtao Li, Yan Ding, Lijuan Wen, Li Wang

**Affiliations:** ^1^CT Section of The Second Hospital Affiliated Qiqihar Medical University, Qiqihar 161000, Heilongjiang, China; ^2^Qiqihar Medical University, Qiqihar 161000, Heilongjiang, China; ^3^Ultrasound Department, The Third Hospital Affiliated Qiqihar Medical University, Qiqihar 161000, Heilongjiang, China; ^4^Radiology Center, The Third Hospital Affiliated Qiqihar Medical University, Qiqihar 161000, Heilongjiang, China

## Abstract

The emergence of energy spectrum CT provides greater diagnostic value for clinical practice. Its advantage is that it can provide more functional imaging parameters and accurate image information for clinical practice, which represents a mainstream direction of CT technology development at present. This paper mainly studies the clinical trial of CAMPO Precision128 Max ENERGY spectrum CT combined with multiple parameters to evaluate the benign and malignant pleural effusion. This paper analyzes the principle and key performance parameters of energy spectrum CT imaging, the etiology of pleural effusion, and its conventional diagnostic methods and uses energy spectrum CT to detect the benign and malignant pleural effusion. In this paper, two groups of patients with different types of pleural effusions were scanned by line spectrum chest CT scans, and energy spectrum analysis software was used to measure and calculate the CT values of conventional mixed energy values of ROI of patients with pleural effusions. For the CT value and energy curve slope measurement value of different single energy keV, independent sample *t*-test was used to analyze and compare the two sets of data, and finally it has been found out that the two sets of data were similar. According to the experimental results, the curves of energy spectrum of the two groups of data are similar in the descending curve of bow-back. The slope of energy spectrum curve in the leakage group was lower than that in the exudate group, showing statistical significance (*P* < 0.05). The slope of energy spectrum curve K in the malignant pleural effusion group was significantly higher than that in the benign pleural effusion group, and the difference was statistically significant (*P* < 0.05). The trend of energy spectrum curves of the two is roughly the same, while at the high energy level, part of the energy spectrum curves of the two are overlapped. The above conclusion indicates that energy spectrum CT plays a certain role in the differential diagnosis of pleural effusion. At the same time, energy spectrum CT also provides a noninvasive and rapid examination method for clinical differentiation of pleural effusion, which has certain clinical application value and prospect.

RETRACTED

## 1. Introduction

In clinical diagnosis of pleural effusion, the existence of pleural effusion should be defined first, then the exudation or leakage of pleural effusion should be distinguished, and finally the specific etiology of pleural effusion should be determined. The presence of pleural effusion should be diagnosed by combining clinical manifestations, physical examination, and instrument examination. Whether pleural effusion is effusion or leakage is mainly identified according to light standard: total protein of pleural effusion/total protein of serum >0.5; lactate dehydrogenase (LDH)/serum LDH > 0.6; lactate dehydrogenase (LDH)/lactate dehydrogenase (LDH) pleural effusion LDH level > serum LDH is 2/3 of the upper limit of normal value. Pleural effusion can be divided into benign pleural effusion (BPE) and malignant pleural effusion (MPE) according to the nature of the etiology [1, 2]. BPE is usually cured by symptomatic treatment, such as anti-infection, antituberculosis treatment, pleura puncture drainage, and closed thoracic drainage. The prognosis is good. Theoretically, all organ malignancies have the possibility of invasion or metastasis to the pleura to cause MPE, including malignant mesothelioma primary cell in the pleura and solid tumors of other organs throughout the body, such as lung cancer, breast cancer, lymphoma, gastrointestinal malignancies, ovarian cancer, and hematological tumors, such as leukemia [3]. The appearance of MPE indicates that the malignant tumor has entered an advanced stage. At this time, the patient clinically presents symptoms such as chest tightness, asthma, and dyspnea, activity endurance is significantly reduced, and the quality of life is seriously decreased. There are significant differences between BPE and MPE in treatment and prognosis. Therefore, accurate differential diagnosis of benign and malignant pleural fluid as soon as possible is of great significance for patients. As a noninvasive method, imaging diagnosis can well show abnormal pleural changes under pathological conditions and provide reliable basis for the diagnosis of clinical pleural effusion.

In clinical work, energy spectrum CT is mainly used in the following clinical work: removal of sclerosing artifacts, quantitative analysis of substances, improving the detection rate of microlesions, qualitative grading of tumors, etc. Many scholars at home and abroad have drawn many conclusions by using energy spectrum CT. According to Rigie's study, the technology of energy spectrum CT to remove metal artifacts can effectively remove the metal artifacts generated after intracranial aneurysm occlusion surgery, more clearly show the intracranial fine structure, and provide strong evidence for the healing of patients. However, his conclusion has not been proved by experiments [4]. According to Danad, the material analysis technique in energy spectrum CT can be used to remove the bone structure and obtain images without calcium content, so as to evaluate the condition of bone marrow. Through the evaluation of the condition of bone marrow, people can predict the damage of bone marrow after bone contusion [5]. However, his study did not involve the detection of thoracic effusion [6]. Danad assessed the blood supply status of fatty liver and liver island by measuring the enhancement rate of iodine (water) concentration in energy spectrum CT, proving that the blood supply status of fatty liver is the same as that of liver island. This is the clinical identification of liver island, providing clinical evidence for the clinical differentiation of liver tumors with deficient blood supply and liver island. However, he did not make a multiparameter comparison [7].

RETRACTED

This paper mainly studied the energy spectrum CT multiparameter joint clinical trials of benign and malignant pleural exudates by collating inductive energy spectrum CT imaging principle and performance parameters, points by spectral imaging technology comprehensive analysis of different performance of benign and malignant pleural effusion, and CT spectral imaging technology in benign pleural effusion and applied value in differential diagnosis of malignant pleural effusion.

## 2. Energy Spectrum CT Evaluation of Pleural Effusion Benign and Malignant Theoretical Basis

### 2.1. Principle and Key Performance Parameters of Energy Spectrum CT Imaging

#### 2.1.1. Principle of Energy Spectrum CT Imaging

Spectral CT imaging is a single instantaneous tube voltage kV switching technology, and the molecular material of gem detector is the core of CT imaging technology [8], energy spectral CT uses a single X-ray tube ball, using 80 rotatekVp and 140 within 0.5 ms kVp fast kVp switch tube voltage rotation, and uses a single tube and a single gem detector to sample two sets of molecular materials to generate dual-energy X-ray imaging [9]. According to the projection of the energy spectrum CT140 kVp low voltage and 80 kVp tube voltage, the selected basic material is mapped to the material density on the projection. The method is to closely combine the material and the projected material density to decompose and generate 101 groups such as keV 40 to 140 keV image. Different materials and different energy levels are matched with the basic material of the decomposition diagram, and the energy spectrum of the CT value that changes with the keV trend curve is generated and used for the quantitative analysis of the effective atomic number of the material. Through the analysis of the lesion, most of the indicators can be obtained, such as imaging information parameters [10].

RETRACTED

#### 2.1.2. Single Energy Imaging

Single molecular material energy imaging is to use gem detector within 0.5 ms through two kV voltage setting (80 kVp and 140 kVp) instantaneous switching between the two groups of data samples, thus generated within 40 keV to 140 keV group level 101 CT images; each organization at each level has a unique CT attenuation characteristics and will organize the relative CT values into absolute CT value. The CT value of each voxel is determined by its mass attenuation coefficient and material density, and the attenuation coefficient is determined by the material type and radiation energy level. Therefore, according to material density, the CT value of each voxel can overlap a variety of material components [11]. Single energy imaging can reflect the X-ray attenuation coefficient of test material to the process of change with the radiation level, checked material in different level of energy level imaging is with different radiation attenuation characteristics, and organization of X-ray attenuation coefficient is different; as a result of the difference in CT values, at lower keV energy levels, the tissue capacity of X-rays is relatively low, while the image noise of the tissue increases. In addition, the X-rays of the tissues are significantly attenuated and the contrast gradually increases. At a high keV energy level, X-rays have a relatively strong ability to penetrate tissues and substances. Single-energy imaging can eliminate image hardening artifacts and improve the noise, but the contrast resolution of tissues also decreases. Under the same single energy condition, the CT value increases gradually with the increase of iodine content, while under the same iodine concentration condition, the CT value decreases gradually with the increase of single energy [12]. Energy spectrum CT can provide single-energy images with different keV, provide more imaging information for disease diagnosis, reduce the hardening artifacts of ray beams and optimize the contrast, and can be used for lesion display, disease diagnosis, and differential diagnosis.

#### 2.1.3. Spectral Curve

Spectrum curve (spectral HU curve) interested in region (region of interest, ROI) within the diseased tissue in different keV imaging with the CT value as keV change trend curve can reflect the CT measurement value of dynamic changes. With the increase of the keV level, different tissue materials under different levels of keV energy spectrum curve have different resolutions and thus produce different spectral curve slope (slope of spectral HU curve, lambda) [13]. For each of the groups, given ROI can automatically generate energy spectrum curve, and according to the increasing number of single keV energy values reflecting the ROI measurement organization dynamic change process of the CT value, it can directly reflect the X-ray absorption differences after penetrating material, showing lesions and normal tissues under the keV energy absorption characteristics. In disease diagnosis and differential diagnosis, multiple lesions homology analysis and group composition identification have a certain application value.

RETRACTED

#### 2.1.4. Separation of Basic Substances

Separation of base material (material decomposition, MD) technology in energy spectrum CT can be any kind of organization of quality into any two kinds of material quality decay, and to achieve with the two substances equivalent of imaging X-ray attenuation, a kind of substance of X-ray attenuation can be converted into two kinds of attenuation. Under the known attenuation level, the mass density and spatial distribution of the substrate are evaluated according to the attenuation degree of the substrate, so as to realize the preliminary analysis of the composition and decomposition. GSI imaging uses fast kVp switching tube voltage system monophyletic double energy scanners to achieve the function base material separation, and according to the effective separation of iodine, fast kVp switching technology base material such as blood, water, fat, calcium, MD, and images can be used for quantitative estimation and measurement of iodine concentration of lesions and normal tissues (iodine concentration, IC), concentration of water (water concentration, WC), and blood concentration (blood concentration, BC). The most commonly used clinical base materials are iodine and water. Iodine substance reaches the lesion through blood circulation, and through quantitative measurement of BC and IC, it can be used to analyze the blood supply of the lesion, observe the curative effect of the disease, and conduct substance quantification.

#### 2.1.5. Effective Atomic Number

Effective atomic number (EFT-Z) is an extension of the concept of atomic number. Based on this principle, the decay characteristic of X-ray can be used to calculate the atomic number of unknown elements. In the application of dual energy subtraction, the DEI (dual energy index) is often used to quantify the energy properties of a substance [14]. DEI is defined as follows:

(1) $$\begin{array}{c} \text{DEI}=\frac{x_{\text{low}}-x_{\text{high}}}{x_{\text{low}}+x_{\text{high}}+2000HU}. \end{array}$$

Physicists came up with the following formula through experiments:

(2) $$\begin{array}{c} \mu \left(E_{1}\right)=f\left(Z^{*},N^{*}\right)N^{*}=\left(AE_{1}^{-m_{2}}{\left(Z^{*}\right)}^{n_{1}}+\sigma \left(E_{1}Z^{*}\right)+BE_{1}^{-m_{2}}{\left(Z^{*}\right)}^{n_{2}}\right)N^{*}, \end{array}$$

where *Z*^*∗*^ is the atomic number of a hypothetical substance. When the X-ray energy level is determined if we simply measure the input X-ray energy and the output X-ray energy, only two variable functions can be obtained. In order to separate the *Z*^*∗*^ value from the above function, energy spectrum technology provides the introduction condition, and another equation is established:

(3) $$\begin{array}{c} \frac{\mu \left(B_{1}\right)}{\mu \left(B_{2}\right)}=\frac{AB_{1}^{-m_{2}}{\left(Z^{*}\right)}^{n_{1}}\sigma \left(B_{1}Z^{*}\right)+BB_{1}^{-m_{2}}{\left(Z^{*}\right)}^{D_{2}}}{AB_{2}^{-m_{1}}{\left(Z^{*}\right)}^{n_{1}}\sigma \left(B_{2}Z^{*}\right)+BB_{2}^{-m_{2}}{\left(Z^{*}\right)}^{D_{2}}}. \end{array}$$

For a pure substance with known components, since its chemical molecular formula is determined, the theoretical value of its effective atomic number can be directly calculated by using the following formula:

(4) $$\begin{array}{c} \text{Eff}-Z=2.94\sqrt{\sum_{i}\left(f_{i}*z_{i}^{2.94}\right)}. \end{array}$$

In clinical applications, the effective atomic number is used to analyze the chemical composition of substances, especially substances with similar density and CT value [15]. Effective atomic number is a new method in CT diagnosis. Currently, it is generally used in the chemical composition analysis of urinary calculi, and it will also be used as one of the parameters in the joint diagnosis of multiple parameters. Its diagnostic value will need to be verified through more clinical research results.

RETRACTED

The extraction of effective atomic number is as follows:

(5) $$\begin{array}{c} \int \frac{\mu_{\tau }\left(E\right)}{\rho_{\tau }}\rho_{\tau }\text{d}s\approx \int \left(\frac{\mu_{\alpha }\left(E\right)}{\rho_{\alpha }}w_{\alpha \tau }+\frac{\mu_{\beta }\left(E\right)}{\rho_{\beta }}w_{\beta \tau }\right)\rho_{\tau }\text{d}s. \end{array}$$

If *T*_1_ and *T*_2_ are used to represent the thickness of the two base materials, then

(6) $$\begin{array}{c} \int \mu_{\tau }\left(E\right)\text{d}s=t_{\alpha }\mu_{\alpha }\left(E\right)+t_{\beta }\mu_{\beta }\left(E\right), \end{array}$$

(7) $$\begin{array}{c} t_{\alpha }=\int \frac{\rho_{\tau }}{\rho_{\alpha }}w_{\alpha \tau }\text{d}s=\frac{\rho_{\tau }}{\rho_{\alpha }}w_{\alpha \tau }t_{\tau }, \end{array}$$

(8) $$\begin{array}{c} t_{\beta }=\int \frac{\rho_{\tau }}{\rho_{\beta }}w_{\beta \tau }\text{d}s=\frac{\rho_{\tau }}{\rho_{\beta }}w_{\beta \tau }t_{\tau }. \end{array}$$

In the perspective system used in this paper, the thickness *t* of the material to be detected is unknown. Therefore, on the basis of the above theory, the following methods are used to extract the effective atomic number:

(9) $$\begin{array}{c} \frac{t_{\beta }}{t_{\alpha }}=\frac{\rho_{\alpha }w_{\beta \tau }}{\rho_{\beta }w_{\alpha \tau }}. \end{array}$$

Finally, the effective atomic number can be obtained as follows:

(10) $$\begin{array}{c} Z_{\tau }^{3.8}=\frac{Z_{\alpha }^{3.8}+C\;\left(t_{\beta }/t_{\alpha }\right)}{1+C\;\left(t_{\beta }/t_{\alpha }\right)}. \end{array}$$

Among them,

(11) $$\begin{array}{c} C=\frac{Z_{\beta }\rho_{\beta }^{2}A_{\alpha }Z_{\beta }^{3.8}}{Z_{\beta }\rho_{\beta }^{2}A_{\alpha }}. \end{array}$$

The attenuation coefficient *T*_*H,L*_ is obtained from high- and low-energy image data:

(12) $$\begin{array}{c} T_{H,L}=-\ln\frac{I}{I_{0}}, \end{array}$$

where *I* is the gray level of the image and *I*_0_ is the empty gray level.

#### 2.1.6. Classification and Evaluation Index of Machine Learning Algorithm

The accuracy of sample data is the ratio of the number of samples correctly classified by the classifier to the total number of samples for a given test dataset. The formula is as follows:

(13) $$\begin{array}{c} A\left(M\right)=\frac{\text{TN}+\text{TP}}{\text{TN}+\text{FP}+\text{FN}+\text{TP}}. \end{array}$$

The accuracy rate is from the perspective of prediction results. The calculation of accuracy rate is the proportion of the predicted results in line with the actual value, which can be understood as the situation without “false alarm,” and the formula is as follows:

(14) $$\begin{array}{c} P\left(M\right)=\frac{\text{TP}}{\text{TP}+\text{FP}}. \end{array}$$

Recall rate is from the perspective of the original sample. The recall rate is calculated as the ratio of the number of correctly classified items to the number of all “should” be correctly classified (in line with the target label), which can be understood as the situation that there is no “missing report” corresponding to the recall rate. The formula is as follows:

(15) $$\begin{array}{c} R\left(M\right)=\frac{\text{TP}}{\text{TP}+\text{FN}}. \end{array}$$

Receiver operating curve (ROC curve) is a graph showing the performance of a classification model under all classification thresholds. This picture depicts two parameters: true positive rate and false positive rate.

RETRACTED

True positive rate TPR is synonymous with the recall rate:

(16) $$\begin{array}{c} \text{TPR}=\frac{\text{TP}}{\text{TP}+\text{FN}}. \end{array}$$

The false positive rate is defined as FPR:

(17) $$\begin{array}{c} \text{FPR}=\frac{\text{FP}}{\text{FP}+\text{TN}}. \end{array}$$

*F*_1_ value is the harmonic mean value of the precision rate and recall rate:

(18) $$\begin{array}{c} \frac{2}{F_{1}}=\frac{1}{P}+\frac{1}{R}, \end{array}$$

namely,

(19) $$\begin{array}{c} F_{1}=\frac{2\text{TP}}{2\text{TP}+\text{FP}+\text{FN}}. \end{array}$$

Regression algorithm indexes include mean absolute deviation, mean square error, *R*^2^ score, and explained variance score.

Average absolute error formula:

(20) $$\begin{array}{c} \text{MAE}=\frac{1}{n}\sum_{i=1}^{n}\left|f_{i}-y_{i}\right|. \end{array}$$

Mean square error formula:

(21) $$\begin{array}{c} \text{MSE}=\frac{1}{n}\sum_{i=1}^{n}{\left(f_{i}-y_{i}\right)}^{2}. \end{array}$$

*R* ^2^ score is the “coefficient of determination,” which is used to judge the fitting degree between the prediction model and the real data. The best value is 1, which can be negative. Assuming that *Y*_*i*_ is the true value and *f*_*i*_ is the corresponding predicted value, the *R*^2^ score of *n* samples is given by the following formula:

(22) $$\begin{array}{c} R^{2}=1-\frac{\sum_{i=1}^{n}{\left(y_{i}-f_{i}\right)}^{2}}{\sum_{i=1}^{n}{\left(y_{i}-\bar{y}\right)}^{2}}, \end{array}$$

where *y* bar is the mean value of *Y*, namely,

(23) $$\begin{array}{c} \bar{y}=\frac{1}{n}\sum_{i=1}^{n}y_{i}. \end{array}$$

Explained variance score: assuming that *y* is the true value, *f* is the corresponding predicted value, and Var is the variance, the explained variance is given by the following formula:

(24) $$\begin{array}{c} \text{Explained Variance}=1-\frac{\text{Var }\left(y-f\right)}{\text{Var }\left(y\right)}. \end{array}$$

The maximum value of the formula is 1, and the closer to 1, the better.

AUC (area under curve) is defined as the area under the ROC curve because the ROC curve is generally above the line *y* = *x*, so the value range is between 0.5 and 1. AUC is used as the evaluation index because the ROC curve cannot clearly indicate which classifier is better, and AUC is a numerical value, and the larger the value, the better the classifier.

The calculation formula of AUC is as follows:

(25) $$\begin{array}{c} \text{AUC}=\frac{\sum_{i\in \text{positive Class}}{\text{rank}}_{i}-\left(M\left(1+M\right)/2\right)}{M\times N}. \end{array}$$

### 2.2. Etiology and Routine Diagnosis of Pleural Effusion

#### 2.2.1. Etiology of Pleural Effusion

Pleural cavity, under normal circumstances, is a closed cavity, in which there is a little liquid. It can play the role of lubrication in the process of breathing, and with a little liquid, it is not always the same. It is a dynamic process, and any disease in the clinical could lead to a dynamic balance is broken, which will be increase in the number of fluid inside the chest, called as a pleural effusion (14 to 15). At present, the qualitative diagnosis of pleural effusion depends on the appearance of observation effusion, routine examination, laboratory examination, imaging examination, detection of tumor markers, tuberculin culture, pleural biopsy [16, 17], fiberoptic bronchoscopy, lymph node biopsy, percutaneous lung biopsy, etc.

RETRACTED

Pleural effusion is classified according to different etiologies. The following are the most common classifications: first, the most traditional classifications of effusion and effusion; second, benign pleural effusion and malignant pleural effusion. It can be divided into malignant pleural effusion (find tumor cells) and tuberculous pleural effusion (find acid-fast bacilli) according to the types of cells contained in pleural water. There are several clinical causes that can lead to pleural effusion, some of which may only lead to pleural effusion and some of which may lead to exudate [18].

#### 2.2.2. Cause of Pleural Effusion

Pleural permeability increases and lining pleural lymphatic is blocked, and chest infective lesions (inflammation and tuberculosis), inflammation of the pleura (tuberculous pleurisy), under the diaphragm inflammation (acute pancreatitis and liver abscess), and chest wall malignant placeholder (chest wall between primary tumors such as leaf tissue source and chest wall tumor metastatic nodules) of these lesions can lead to pleural exudate. Neoplastic lesions can lead to lymphatic obstruction and pleural effusion, and abnormal lymphatic drainage during development can also lead to pleural effusion. Iatrogenic diseases and injuries can also cause exudation or leakage of fluid. Aortic aneurysm or aortic dissection can cause bloody hydrothorax and perforation of the esophagus in advanced esophageal cancer may cause empyema; if the thoracic duct is ruptured, it will lead to chylothorax [19]. Some clinical drugs (amiodarone and furantoin), surgical operations (radiotherapy, endoscopy, coronary artery bypass grafting, and stent implantation), and peritoneal dialysis may all cause effusion.

#### 2.2.3. Biochemical Examination of Pleural Effusion

In the past, the pleural effusion was mainly distinguished by its appearance, cells in the pleural effusion, PH value, glucose, pathogen, protein, and enzyme content. If the color of the liquid is transparent and has no odor, it can be considered as leaking liquid. If the color of the liquid is dark and sometimes yellow with turbidity, coagulation can occur after standing, and it is preliminarily judged as exudate. The division standard according to the proportion is bounded (1.018), the content of protein is 30 g/L, and the number of white blood cells is 500 × 10^6^/L, less than the above numerical upper bound for the leaking liquid, whereas for the exudate, the index in pleural effusion and leakage of liquid in the differential diagnosis of its sensitivity and specific degree is not high, so the clinical work rarely used the standard [20]. At present, serous cavity effusion is mainly divided into exudate and leakage fluid according to the light standard. The sensitivity and specificity of this standard in diagnosing exudate are about 96% and 80%, respectively. Although the light standard has a high sensitivity, it does not have a high specificity in diagnosing exudate.

RETRACTED

#### 2.2.4. Conventional Diagnostic Methods

The gold standard for the qualitative diagnosis of pleural effusion is pleural puncture and drainage. X-ray chest film, B-ultrasound examination, conventional CT examination, and energy spectrum CT examination are the most commonly used imaging methods for the diagnosis of pleural effusion. With the development of science and technology, the imaging diagnosis method has the advantages of simple operation, noninvasive, and rapid. It has been gradually applied in the differential diagnosis of pleural effusion. It can not only determine whether there is pleural effusion but also determine the cause and nature of pleural effusion through indirect signs such as chest and pleura [21].

### 2.3. Qualitative Value of Energy Spectrum CT in Benign and Malignant Pleural Effusion

#### 2.3.1. The Value of Single Energy CT in Differentiating Benign Pleural Effusion from Malignant Pleural Effusion

During the implementation of energy spectrum CT scanning, two sets of data were obtained through the instantaneous conversion of high and low energy of 80 kVp and 140 kVp. After the spatial projection analysis of the two sets of original data, a series of single-energy images from 40 keV to 140 keV could be obtained. A single energy image represents a specific level of X-ray attenuation. Low-energy X-rays exhibiting different characteristics at different energy levels have a weaker passing ability. As the image level increases the resolution of the tissue, the noise will increase. Utilizing the power of high-energy X-rays, the level of the image can reduce hardening artifacts but weaken the contrast between tissue resolutions. For a single energy image at the same level, the absorption coefficient of a substance is determined by its own density, so as to ensure the consistency of the material attenuation coefficient of the same organizational structure, avoid the generation of hardening artifacts, and obtain accurate CT value [22, 23]. The main components of benign and malignant pleural effusion include protein content, cell count, blood fine clot, and enzyme content .The CT values of benign and malignant pleural effusions are significantly different at different single energy levels. When the energy level is lower, the difference in CT values between the two groups is more prominent, especially at a single 40 keV energy level. Comparing the CT values of the two groups, the 40 keV~80 keV energy level of the CT values of malignant pleural effusion was significantly higher than that of the benign pleural effusion group. As the keV value increases, the difference in CT values of benign and malignant pleural effusions is decreasing, and there is a partial overlap. This is corresponding to the principle of energy spectrum imaging. The tissue contrast of high-energy images is relatively weak, while that of low-energy images is obviously related, which indicates that the difference of tissue chemical composition in substances can be better reflected by using the low energy level.

RETRACTED

Single energy, according to the optimization of organizational structure in contrast from another point of view, shows the organizational structure of the different components better; low energy levels are beneficial to enhance the visibility of the organizations and travel is much easier to show the opposite sex, thus improving the detection of small lesions or ingredients within the organizational structure which has the different components [24].

#### 2.3.2. The Value of Energy Spectrum Attenuation Curve in Differential Diagnosis of Benign Pleural Effusion and Malignant Pleural Effusion

The basic principle of energy spectrum CT imaging is that different objects have different X-ray attenuation characteristics for different energy levels. The absorption curve of a substance represents the attenuation of X-rays after passing through a certain substance, which can be used at different single energy (keV). For the average CT value, it depends on the chemical composition of the substance that the tissue structure of various substances is different, and each has a different absorption attenuation curve with a different CT value. Therefore, different attenuation curves are used to evaluate the difference in the chemical composition of materials, and the difference in the attenuation curve is mainly quantitatively evaluated by the slope of the curve [25]. Energy spectrum CT imaging can obtain a series of single-energy images, and each energy level has a relatively accurate CT value, so as to obtain the corresponding energy spectrum curve. At low energy levels (40 keV–80 keV), spectrum curve of the slope in different effusions have significant differences, and vicious decline is more apparent than the benign group. In the low energy levels, the spectral curve slope of change seems to be more intuitive, so the metabolites in benign and malignant pleural effusion and chemical composition are different, and in 90 keV–140 keV energy levels, different curve lines gradually flatten out, almost overlapping part of the curve in high energy level, and CT value also increased with the increase of energy to reduce gradually between the energy levels of two groups of effusion, making little sense to identify [26, 27].

RETRACTED

## 3. Application of Energy Spectrum CT in Evaluating Benign and Malignant Pleural Effusion

### 3.1. Selection of Research Objects

The subjects of this study were 50 patients who were clinically diagnosed with pleural effusion and underwent pleural effusion biochemical examination in our hospital in the last year. By routine pleural effusion and biochemical examination, according to standards such as light, 50 patients were divided into the exudate group and the leakage group, among which the exudate group was further divided into benign pleural effusion and malignant pleural effusion. As shown in Table 1, the basic information of patients is shown in Table 1.

### 3.2. Selection Criteria and Exclusion Criteria of Research Objects

#### 3.2.1. Selection Criteria

Patients admitted were to our hospital and clinically diagnosed as pleural effusion. The patients underwent pleural fluid biochemical examination and were diagnosed as exudate or leakage fluid in our hospital. Plain chest scan by energy spectrum CT was performed in the CT room of our hospital. Patients could cooperate to complete the examination. The amount of pleural effusion reached medium or large amount, and the images met the quality requirements.

#### 3.2.2. Exclusion Criteria

After the completion of energy spectrum CT scan, the amount of pleural effusion was too small, which was not conducive to the measurement of the operator, and the relevant indexes cannot be measured and calculated. During the scanning process, the patient had poor cooperation, the respiratory artifact and motion artifact were large, the image quality was poor, and the patient had claustrophobia and cannot be examined. The patients were clinically diagnosed as pleural effusion and did not receive energy spectrum CT chest plain scan or biochemical examination of pleural effusion.

RETRACTED

### 3.3. Content and Method of the Research

#### 3.3.1. Image Acquisition

Plain chest CT scan was performed using CAMPO Precision128 Max energy spectrum CT mode. Before the examination, the patient's breathing was trained to reduce respiratory artifacts, so as to successfully complete the scan and sign the informed consent. The patient was placed on the back and scanned from the thoracic entrance to the entire lung field at the diaphragmatic top.

#### 3.3.2. Image Analysis

Image analysis was carried out using spectral analysis software on the workstation AW4.6 start viewer software, and the three most important pleural effusion layers used to measure ROI were selected; in this experiment, we measured the level of each selected three interested area (ROI) and obtained the average of the three points; then, the three levels of three average sum end up with an average. In the selection of measurement points, the location with deep effusion should be chosen as far as possible to avoid necrotic and atelectatic lung tissue, reduce the influence of artifact artifacts, and stay away from bony structures such as ribs and spine. 40–140 kev AW4.6 postprocessing software was used to automatically generate an image of a single energy spectrum images and matching base material (iodine-water and water-iodine diagram), record the ROI measurement under CT value, effective atomic number, and single energy matching base material, take on a level three average, calculate the average of three planes, and then analyse the image data.

### 3.4. Statistical Method

SPSS22.0 statistical software was used for analysis. The characteristic parameters of energy spectrum of exudate and leakage fluid were compared: the data of each group were consistent with the normal. For the data of two independent samples, independent sample *T* should be used to check whether the data of the two groups were different and whether they were statistically significant (*P* < 0.05). The CT values of benign pleural effusion and malignant pleural effusion at different energy levels of 40–140 keV were analyzed, and the slope of energy spectrum curves of benign pleural effusion and malignant pleural effusion were compared using the Mann–Whitney test. The Mann–Whitney test was used to compare the CT values of benign pleural effusion and malignant pleural effusion at the conventional mixed energy level. *P* < 0.05 was considered statistically significant.

## 4. Application of Energy Spectrum CT in Evaluating Benign and Malignant Pleural Effusion

### 4.1. CT Value Comparison of Mixed Energy of Exudate and Leakage Fluid

As shown in Table 2 and Figure 1, the minimum CT value and maximum CT value under the mixed energy of leakage fluid are 9.23 and 13.07, respectively. Under the mixed energy of exudate, the minimum CT value was 16.15 and the maximum value was 22.40. The *T* value was –7.731, *P* < 0.05, indicating that the data of the two groups were different and statistically significant (*P* < 0.05).

RETRACTED

### 4.2. Comparison of Slope of Exudate Curve and Leakage Curve

As shown in Table 3 and Figure 2, in benign pleural effusion, the levels of ADA and CRP were higher than those in malignant pleural effusion, and the levels of LDH and CEA were lower than those in malignant pleural effusion. The difference between the two groups was statistically significant (*P* < 0.01).

### 4.3. Comparison of Slope of Energy Spectrum Curve between Malignant Pleural Effusion and Benign Pleural Effusion

The maximum, minimum, and median values of postoperative total fluid recovery time of patients in the three groups, same as the previous two statistical indicators of patients, were still selected.

As shown in Table 4 and Figure 3, the positive rates of ADA and CRP in benign pleural effusion group were higher than those in malignant pleural effusion group, and the positive rates of LDH and CEA in benign pleural effusion group were lower than those in malignant pleural effusion group. The difference between the two groups was statistically significant (*P* < 0.01).

### 4.4. CT Value Analysis of Malignant Pleural Effusion and Benign Pleural Effusion under Different keV

According to Table 5 and Figure 4, the lower the CT value of benign and malignant pleural effusion at different single energy levels, the more obvious the difference between the two groups, especially at the 40VkeV energy level in a single group, the difference between the two is most obvious. When the CT values of the two groups were between 40 keV and 80 keV, the CT values of the malignant pleural effusion group were significantly higher than those of the benign pleural effusion group, and the difference was statistically significant.

As shown in Table 6 and Figure 5, there were significant differences in CT values of 40 keV and 100 keV single energy images between benign and malignant pleural effusions (all *P* < 0.001), and significant differences in effective atomic number (*P* < 0.05).

### 4.5. CT Value Comparison of Malignant Pleural Effusion and Benign Pleural Effusion under Conventional Mixed Energy

As shown in Table 7 and Figure 6, there was no significant difference in the slope of energy spectrum curve, CT value of mixed energy image, water base value, lipid base value, and blood base value between benign and malignant pleural effusion (all *P* < 0.05).

RETRACTED

## 5. Conclusions

Pleural effusion (PE) is a very common disease. Due to its multiple and complex etiologies and different pathogenesis, invasive methods are often required for diagnosis. It has been reported that the manifestations of tuberculous pleurisy and malignant pleural effusion are mainly lymphocytes, and the routine and biochemical results are often similar. In view of the great difference in treatment and prognosis between tuberculous pleural effusion (TPE) and malignant pleural effusion (MPE), early differential diagnosis is particularly important. The innovation of this paper is to fully consider the advantages and disadvantages of spectral CT, highlight its role in the diagnosis of benign and malignant pleural effusion, and emphasize its breakthrough in practical application.

This article uses CT spectral imaging technology to observe the CT value and the change of the spectral curve slope of benign pleural effusion and malignant pleural effusion, and compare the difference of conventional mixed energy under two kinds of CT. According to the comprehensive analysis of the comprehensive value of spectrum imaging technology for benign and malignant pleural effusion, the application value of energy spectrum CT imaging technology in the identification of benign pleural effusion and the differential diagnosis of malignant pleural effusion is obtained..

In this study, by analyzing the multiparameter images of the exudate group and the leakage group, the CT value under mixed energy and the CT value under single energy were compared with each other in terms of the slope of energy spectrum curve, among which the difference of the slope of the energy spectrum curve was more obvious. The above conclusion indicates that energy spectrum CT plays a certain role in the differential diagnosis of pleural effusion. At the same time, energy spectrum CT also provides a noninvasive and rapid examination method for clinical differentiation of pleural effusion, which has certain clinical application value and prospect.

## Figures and Tables

**Figure 1:** Comparison of the CT value under mixed energy of pleural effusion in two groups.

**Figure 2:** Comparison of various indexes in benign and malignant pleural effusion.

**Figure 3:** Comparison of positive rates of four indexes in benign and malignant pleural effusion.

**Figure 4:** Comparison of the CT value between benign and malignant pleural effusion from 40 keV to 130 keV.

**Figure 5:** Comparison of related parameters of energy spectrum CT in benign and malignant pleural effusion.

**Figure 6:** Comparison of the CT value of benign and malignant pleural effusion under conventional mixed energy.

RETRACTED

**Table 1:** Basic information of patients.

Group	Sex ratio (male : female)	*N*	Age	Weight
All patients	27 : 23	50	61.8 ± 6.37	57.19 ± 7.24
Benign exudate	12 : 9	21	60.9 ± 6.25	59.36 ± 7.15
Malignant exudate	9 : 10	19	60.4 ± 6.52	56.27 ± 7.06

**Table 2:** Comparison of the CT value under mixed energy of pleural effusion in two groups.

CT value	1	2	3	4	5	6
Leakage fluid	9.23	10.27	11.14	11.21	12.16	13.07
Exudate	16.15	17.71	18.96	19.57	20.83	22.40

**Table 3:** Comparison of various indexes in benign and malignant pleural effusion.

Group	ADA (U/L)	CRP (mg/L)	LDH (U/L)	CEA (ug/L)
Benign	61.1 ± 10.2	23.7 ± 5.4	442.8 ± 110.2	8.4 ± 1.2
Malignant	15.5 ± 5.2	4.6 ± 2.2	961.1 ± 212.9	21.6 ± 11.7
*T* value	8.33	6.78	9.23	8.97
*P* value	<0.01	<0.01	<0.01	<0.01

**Table 4:** Comparison of positive rates of four indexes in benign and malignant pleural effusion.

Group	ADA (U/L)	CRP (mg/L)	LDH (U/L)	CEA (ug/L)
Benign	170	171	20	5
Malignant	6	8	37	35
*X* ^2^ value	11.56	24.66	5.21	7.87
*P* value	<0.01	<0.01	<0.01	<0.01

**Table 5:** Comparison of the CT value between benign and malignant pleural effusion from 40 keV to 130 keV.

	40 keV	50 keV	60 keV	70 keV	80 keV	90 keV	100 keV	110 keV	120 keV	130 keV
Benign	17.84	15.62	14.20	13.47	12.93	12.54	12.26	12.02	11.93	11.82
Malignant	47.51	34.43	26.19	20.62	17.49	15.23	13.91	13.07	12.04	11.46

**Table 6:** Comparison of related parameters of energy spectrum CT in benign and malignant pleural effusion.

Nature of effusion	CT value of mixed energy image (HU)	Slope of energy spectrum curve	CT value of 40 keV single energy image (HU)	CT value of 100 keV single energy image (HU)
Benign	12.61 ± 3.39	0.56 ± 0.04	43.15 ± 3.79	9.11 ± 1.38
Malignant	14.71 ± 5.03	0.59 ± 0.04	39.42 ± 2.60	6.52 ± 2.04
*T* value	0.200	0.057	0.005	<0.001

**Table 7:** Comparison of the CT value of benign and malignant pleural effusion under conventional mixed energy.

	Water base value (mg/cm^3^)	Aliphatic value (mg/cm^3^)	Blood base value (mg/cm^3^)	Effective atomic number
Benign	1016.90 ± 19.83	–379.70 ± 38.68	1625.3 ± 98.44	7.87 ± 0.08
Malignant	1008.41 ± 12.22	–392.60 ± 41.28	1655.8 ± 106.24	7.90 ± 0.02
*T* value	0.180	0.390	0.430	0.020

## Data Availability

No data were used to support this study.

## References

[1] Weick J. K., Kiely J. M., Harrison E. G. (2015). Pleural effusion in lymphoma. *Cancer*.

[2] Fentiman I. S., Millis R., Sexton S. (2015). Pleural effusion in breast cancer: a review of 105 cases. *Cancer*.

[3] Zhao Y., Li H., Wan S. (2019). Knowledge-aided convolutional neural network for small organ segmentation. *IEEE Journal of Biomedical and Health Informatics*.

RETRACTED

[4] Rigie D. S., La Rivière P. J., Patrick J. (2015). Joint reconstruction of multi-channel, spectral CT data via constrained total nuclear variation minimization. *Physics in Medicine and Biology*.

[5] Song H., Brandt-Pearce M. (2013). Range of influence and impact of physical impairments in long-haul DWDM systems. *Journal of Lightwave Technology*.

[6] Danad I., Fayad Z. A., Willemink M. J., Min J. K. (2015). New applications of cardiac computed tomography: dual-energy, spectral, and molecular CT imaging. *JACC: Cardiovascular Imaging*.

[7] Zimmerman K. C., Schmidt T. G. (2015). Experimental comparison of empirical material decomposition methods for spectral CT. *Physics in Medicine and Biology*.

[8] Zhao Y., Zhao X., Zhang P. (2015). An extended algebraic reconstruction technique (E-ART) for dual spectral CT. *IEEE Transactions on Medical Imaging*.

[9] Zhang Y., Xi Y., Yang Q., Cong W., Zhou J., Wang G. (2016). Spectral CT reconstruction with image sparsity and spectral mean. *IEEE Transactions on Computational Imaging*.

[10] Foygel Barber R., Sidky E. Y., Gilat Schmidt T., Pan X. (2016). An algorithm for constrained one-step inversion of spectral CT data. *Physics in Medicine and Biology*.

[11] Liu H., Yan F., Pan Z. (2015). Evaluation of dual energy spectral CT in differentiating metastatic from non-metastatic lymph nodes in rectal cancer: initial experience. *European Journal of Radiology*.

[12] Li C., Shi C., Zhang H., Hui C., Lam K. M., Zhang S. (2015). Computer-Aided diagnosis for preoperative invasion depth of gastric cancer with dual-energy spectral CT imaging. *Academic Radiology*.

[13] Li G. J., Gao J., Wang G. L., Zhang C. Q., Shi H., Deng K. (2016). Correlation between vascular endothelial growth factor and quantitative dual-energy spectral CT in non-small-cell lung cancer. *Clinical Radiology*.

[14] Inyoung S., Geun Y. J., Hee P. J. (2016). Virtual non-contrast CT using dual-energy spectral CT: feasibility of coronary artery calcium scoring. *Korean Journal of Radiology*.

[15] Li L., Chen Z., Cong W., Wang G. (2015). Spectral CT modeling and reconstruction with hybrid detectors in dynamic-threshold-based counting and integrating modes. *IEEE Transactions on Medical Imaging*.

[16] Raju R. N., Kardinal C. G. (2015). Pleural effusion in breast carcinoma: analysis of 122 cases. *Cancer*.

[17] Elis A., Blickstein D., Mulchanov I. (2015). Pleural effusion in patients with non-Hodgkin’s lymphoma: a case-controlled study. *Cancer*.

[18] Seman G., Hunter S. J., Miller R. C., Dmochowski L. (2015). Characterization of an established cell line (SH-3) derived from pleural effusion of patient with breast cancer. *Cancer*.

[19] Kugelman A., Gonen R., Bader D. (2015). Potential role of high-frequency ventilation in the treatment of severe congenital pleural effusion. *Pediatric Pulmonology*.

RETRACTED

[20] Chan G. M., Lechtenberg E. (2015). The use of fat-free human milk in infants with chylous pleural effusion. *Journal of Perinatology*.

[21] Madan K., Mohan A., Hadda V. (2015). Utility of semi-rigid thoracoscopy in undiagnosed exudative pleural effusion. *Lung India*.

[22] Rakvongthai Y., Worstell W., El Fakhri G., Bian J., Lorsakul A., Ouyang J. (2015). Spectral CT using multiple balanced *K*-edge filters. *IEEE Transactions on Medical Imaging*.

[23] Schmidt T. G., Zimmerman K. C., Sidky E. Y. (2015). The effects of extending the spectral information acquired by a photon-counting detector for spectral CT. *Physics in Medicine and Biology*.

[24] Liu L., Zhi X., Liu B., Zhang Y. (2016). Utilizing gemstone spectral CT imaging to evaluate the therapeutic efficacy of radiofrequency ablation in lung cancer. *La Radiologia Medica*.

[25] Takagi H., Murata I. (2016). Development of precise energy spectrum measurement technique for high-power pulsed X-ray sources for industrial use. *Journal of Nuclear Ence and Technology*.

[26] Li L., Wang F., Shang F., Jia Y., Zhao C., Kong D. (2017). Energy spectrum analysis of blast waves based on an improved Hilbert-Huang transform. *Shock Waves*.

[27] Eddrief M., Marangolo M., Etgens V. H. (2006). Interface bonding of a ferromagnetic/semiconductor junction: a photoemission study of Fe/ZnSe (001). *Physical Review B*.

